This article has been retracted.

# α-bisabolol enhances radiotherapy-induced apoptosis in endometrial cancer cells by reducing the effect of XIAP on inhibiting caspase-3

**DOI:** 10.1042/BSR20190696

**Published:** 2019-06-10

**Authors:** Dongmei Fang, Hongxin Wang, Min Li, Wenwen Wei

**Affiliations:** Department of Gynecology, The Second Children and Women’s Healthcare of Jinan City, Jinan, Shandong 271100, China

**Keywords:** α-bisabolol, apoptosis, endometrial cancer, radiotherapy, XIAP/ caspase-3 pathway

## Abstract

Endometrial cancer (EC) is one of the most common cancers in females. Although the diagnosis and treatment in early stages can greatly improve the survival rate of patients, the advanced EC still is lethal. Radiotherapy is widely used against EC, and it is a great challenge to find an effective way to overcome the resistance of EC during radiotherapy. α-bisabolol is a promising drug, which has already exhibited its anti-tumor effect in some malignancies. Here we reported that α-bisabolol could inhibit the proliferation of EC cells. It is also shown that their abilities of migration and invasion were effectively reduced by α-bisabolol. Furthermore, our results also demonstrated that α-bisabolol could improve sensitivity of EC cells in radiotherapy and further inhibited the growth of EC cells. By Western blot, we found the expression of matrix metalloproteinases-9 (MMP-9) and cyclin E were significantly decreased, which indicated that EC cells can be further suppressed by using α-bisabolol and radiotherapy. It is also demonstrated in our study that the rate of apoptotic cells is markedly increased in EC by using these two treatments. The significant decrease in X-linked inhibitor of apoptosis protein (XIAP) and increase in caspase-3 detected in our study suggested that the enhancement of apoptosis is mediated by XIAP/caspase-3 pathway, which was further confirmed by examining the downstream effectors of caspase-3, COX-2, PARP and cleaved PARP. In the present study, we demonstrated that α-bisabolol could enhance the sensitivity of EC cells to radiotherapy, which provide a novel alternative for overcoming radioresistance of EC cells and achieving a better outcome in radiotherapy.

## Introduction

Endometrial cancer is (EC) the most frequent malignancy diagnosed in women [1–4]. The incidence of EC has shown an increasing trend in recent years [5]. There were 288000 new patients diagnosed with this kind of malignancy just in 2008. In North America and Europe, it is the fourth most common female malignancy, and the EC patients’ age become younger [6]. Most patients with EC are diagnosed in stages I or II, the early stages, and its 5-year survival rate is up to 91%. For female with advanced EC (stage III or IV), the 5-year survival rates range from 20 to 66%. Because of the frequent recurrence in the treatment of advanced EC, the patients are usually at a high risk of death [7–10].

Chemotherapy and radiotherapy are always considered as efficient treatments, while the resistance of cancers becomes a barrier. Many studies reported that the resistance of cancers involves some important genes, like matrix metalloproteinases-9 (MMP-9) and cyclin E, which are strongly related to biological properties of cancer cells, such as proliferation, migration and invasion. MMP-9 is a 92-kDa protein, which can degrade some extracellular matrix macromolecules (elastin, laminin, collagen etc.) and basement membrane to promote metastasis and invasion of various carcinomas [11,12]. Cyclin E is a key protein to regulate the transition of cells from G_1_ to S phase. It contributes to unrestricted proliferation of cancer cells via controlling RB pathway [13–15]. Thus, the deregulation of cyclin E usually is linked to various malignancies, for example, lung, breast, ovarian or endometrial cancer [14,16–18].

Apoptosis, a kind of programmed cell death, is a mechanism to eliminate harmful or redundant cells and maintain stability in organizations. Therefore, it is employed during radiotherapy to kill cancer cells. As key factors, caspases are involved in the initiation and execution of apoptosis [19]. Caspase-3 is a type of executioner caspase, which can proteolyze a lot of substrates causing the death of cell [20], while its direct inhibitor, X-linked inhibitor of apoptosis protein (XIAP), can prevent cell from apoptosis by suppressing caspase cascade [21]. Thus, XIAP/caspase-3 pathway may play an important role in radiotherapy-induced apoptosis. COX-2 and PARP are downstream effectors of caspase-3. It is shown that COX-2 was inhibited by caspase-3 after irradiation, and the inhibition of COX-2 could sensitize cancer cells to apoptosis [22,23]. RAPR is another important substrate of caspase-3, in which it is decomposed to an 85-kDa product, cRAPR, that can be identified as an apoptotic marker [24–26].

α-bisabolol is an oily sesquiterpene alcohol [27,28], which is widely derived from several kinds of plants (e.g. *Matricaria recutita*, Myrtaceae, Lamiaceae and Apiaceae) [29–32]. α-bisabolol has multi-functions, such as antimicrobial, anti-inflammatory, anti-nociceptive and even anti-cancer activities [27,28,33]. Besides, it was shown that α-bisabolol attenuated inflammatory response by down-regulating the expression of COX-2 in RAW264.7 macrophages [34]. There are also various studies demonstrating the inhibitory effect of α-bisabolol in glioma, liver carcinoma, acute leukemia and pancreatic cancer [35–38]. However, its anti-cancer activity in EC still remains unknown.

In the present study, we confirmed the anti-cancer effect of α-bisabolol in EC and investigate its potential to enhance sensitivity of EC cells to radiotherapy. Out results also demonstrated that α-bisabolol significantly reduced the expression of MMP-9 and cyclin E during radiotherapy, which further suppressed cancer cells. Furthermore, it is shown in our study that the enhancement of killing effect of radiotherapy with α-bisabolol is mediated by XIAP/caspase-3 pathway in apoptosis. Those results indicated α-bisabolol’s great potential as an adjuvant therapy in the clinical treatment of EC.

## Materials and methods

### Cell culture

EC cell lines including RL95-2, ECC001 and ECC003 cells were purchased from China Center for Type Culture Collection (CCTCC, Wuhan, China). Ishikawa cell line was purchased from European Collection of Authenticated Cell Cultures (ECACC, Salisbury, U.K.). ECC-E6/E7 cell line was obtained from Gynecological Tumor Laboratory of China Medical University. Dulbecco’s modified Eagle’s medium (DMEM) and 0.25% trypsin were purchased from Gibco (Thermo Fisher Scientific, Waltham, U.S.A.). RL95-2, ECC001, ECC003 and Ishikawa cells were cultured in DMEM and ECC-E6/E7 cell was cultured in DMEM/F12 (DMEM:F12 = 1:1). Besides, all cells were cultured with 10% fetal bovine serum (Biological Industries, Cromwell, U.S.A.) and Penicilillin (100 U/ml) and Streptomycin (100 μg/ml) from HyClone (Thermo Fisher Scientific, Waltham, U.S.A.) under 5% CO_2_ in the incubator at 37°C.

### Cell viability assay and clonogenic assay

ATPlite luminescence assay system (PerkinElmer, Waltham, U.S.A.) was used to detect the viability of EC cells. Experiment was carried out following the instructions. Different concentrations of α-bisabolol (purity: ≥ 95%, Sigma, Saint Louis, Missouri, U.S.A.) was used in the experiment, independently. The half-maximal effective concentration (EC_50_) and the half-maximal lethal concentration (LC_50_) values were calculated by Compusyn software with the dose–response curves. For clonogenic assay, cells were digested and resuspended in six-well cell culture plates (Corning-Costar, New York, U.S.A.). Crystal Violet was employed and the number of colonies were counted.

### Wound-healing migration and transwell invasion assay

RL95-2, ECC001 cells were selected for the assays. Briefly, for wound-healing migration assay, cells were grown in six-well cell culture plates to 80% confluence and were then wounded. Optical microscope was used to calculate the ratio of cells that grew in the wounded area. Twenty-four-well Boyden chamber with a non-coated 8-mm pore size filter in the insert chamber (BD Falcon, Corning-Costar, New York, NY, U.S.A.) was used for transwell invasion assay. The two sides of chamber contained with cell culture medium with or without FBS, and cells were cultured for 24 h to test percentage of invasion cells.

### Detection of apoptosis

RL95-2 cells were treated with radiotherapy, α-bisabolol or the coordination of both. Hoechst Staining Kit (C0003) was purchased from Beyotime (Shanghai, China) to detect the apoptotic cells. Experiment was carried out according to the instructions.

### Western blot analysis

Anti-COX2/Cyclooxygenase 2 antibody (ab179800), anti-Cleaved PARP1 antibody (ab32561), anti-PARP antibody (ab74290), anti-XIAP antibody (ab21278), anti-MMP9 antibody (ab73734), anti-Cyclin E1 antibody (ab33911) and anti-GAPDH antibody (ab181602) were purchased from Abcam (Cambridge, U.K.) and were used as primary antibodies. Proteins were collected on ice using NP40 cell lysis buffer for 30 min and then were separated by 8% sodium dodecyl sulfate/polyacrylamide gel electrophoresis (SDS/PAGE). Then the gel was transferred on to polyvinylidene difluoride (PVDF) membrane for 2 h. Five percent milk-TBST (TBS with 0.05% Tween 20) was used for 1 h to block membrane and then was incubated with specific primary antibodies overnight at 4°C. Before incubated by secondary antibody for 1.5 h, the membrane was washed by TBST. ECL reagent was used to visualize proteins and ImageJ software was used to analyze the obtained data.

### Statistical analysis

GraphPad and SPSS 25.0 were used for the data. All experiments were repeated at least three times independently. *P*-value that represents for significant difference was evaluated by two-tailed *t* test (*P<0.05, **P<0.01).

## Results

### α-bisabolol inhibits the growth of EC

To investigate the anti-cancer effect of α-bisabolol in EC, five EC lines were selected comparing with ECC-E6/E7, and dose–response assays were carried out with α-bisabolol treatment for 24 h. By analyzing the rate viability rate, we found significant differences in the sensitivity between EC lines and control to α-bisabolol with the concentrations ranging from 4 to 16 μmol/l (Figure 1A). The result exhibited the anti-cancer effect of α-bisabolol on EC and indicated that EC lines were more sensitive to α-bisabolol. The EC_50_ and the LC_50_ were also consistent with these conclusions. The average values of EC_50_ and LC_50_ were 7.9 and 3.4 in EC cells, respectively, which were markedly smaller than that of control (18.7 of EC_50_ and 4.9 of LC_50_) (Figure 1B).

**Figure 1:** The influence of α-bisabolol on the viability of EC cells (**A**) Dose–response assays. EC cells were treated with different concentrations (from 0 to 32 μmol/l) of α-bisabolol for 24 h, and ECC-E6/E7 was used as the control. Three experiments were performed independently, and ±STDEV was shown with each value. (**B**) Analysis of EC_50 _and LC_50_. STDEV, Standard Deviation.

### The migration and invasion of EC cells were decreased by using α-bisabolol

To further explore the potential of α-bisabolol on the treatment for EC, we performed wound-healing migration assays with two EC lines, RL95-2 and ECC001. For determining biological function of α-bisabolol on cancer cells, a concentration of 4 μmol/l was selected, which could kill approximately 20% ( RL95-2) or 25% (ECC001) of cancer cells. According to our results, only 31% (RL95-2) and 21.5% (ECC001) of width in control’s wound was left after 24 h on average, while that in EC lines was 68.5% (RL95-2) and 42% (ECC001) (Figure 2A).

**Figure 2:** α-bisabolol inhibits the migration and invasion of L95-2 and ECC001 cell lines Wound healing assays (**A**) and transwell invasion assays (**B**) were carried out with RL95-2 and ECC001, respectively. The assays were performed with α-bisabolol in 4 μmol/l for 24 h. Three experiments were performed independently, and ±STDEV was shown with each value, **P<0.01.

In addition to migration, we also determined the change of invasion ability of EC cells. Transwell invasion assay was carried out, and the invasion of cancer cells was measured after 24 h. Comparing with the control that was without the treatment of α-bisabolol, the invasion ability of EC cells were reduced to approximately 57.5 and 27% in RL95-2 and ECC001, respectively (Figure 2B). All these results above demonstrated that α-bisabolol could efficiently impair the migration and invasion abilities of EC cells, indicating its potential as an anti-cancer drug.

### α-bisabolol exhibits a synergistic effect with radiotherapy against EC

We also investigated the effect of radiotherapy on EC cells in combination with α-bisabolol. The results of clonogenic assays showed that the combination of α-bisabolol and radiotherapy can achieve a better inhibitory outcome (23% on average) though that of irradiation (43% on average) was stronger than that of α-bisabolol (70% on average) (Figure 3A). Our results of dose–response assays suggested that there was an enhancement of radiosensitivity induced by α-bisabolol in this combination (Figure 3B), in which EC cells were more sensitive when the dose of irradiation was between 2 and 8 Gy. The EC_50_ and LC_50_ of EC cells were markedly reduced (from 7.45 to 5.65 in EC_50_; from 4.85 to 3.0 in LC_50_), which were consistent with the results above (Figure 3C). For further confirming this conclusion, we also detected two biomarkers of EC, MMP-9 and cyclin E. It is shown in our data that the expression of MMP-9 and cyclin E was significantly decreased (Figure 3D). These results were consistent with previous studies and proved that the EC cells were substantially suppressed with α-bisabolol and radiotherapy.

**Figure 3:** Effect of radiotherapy on EC cells in combination with α-bisabolol (**A**) Clonogenic assays in RL95-2 and ECC001. The cells were treated with α-bisabolol (4 μmol/l), radiotherapy (4 Gy) or the combination of α-bisabolol and radiotherapy for 24 h, respectively, and then the colonies were measured. Three experiments were performed independently, and ±STDEV was shown with each value, **P<0.01. The viability rate (**B**), EC_50_ and LC_50_ (**C**) of RL95-2 and ECC001 are analyzed from three independent experiments of dose–response assays; ±STDEV was shown with each value. (**D**) Western blot analysis for MMP-9 and cyclin E protein in EC cells. GAPDH was used as the loading control. Three experiments were performed independently, and ±STDEV was shown with each value, *P<0.05 and **P<0.01.

### α-bisabolol promotes apoptosis by XIAP/caspase-3 pathway in radiotherapy

Since inducing apoptosis is the main way to kill cancer cells in radiotherapy, we determined the apoptotic rates in different treatments. Via Hoechst 33258 staining, it is exhibited that the apoptotic rate of EC cells was greatly increased when combining irradiation and α-bisabolol, which nearly doubled that of only irradiation or α-bisabolol (Figure 4A).

**Figure 4:** Apoptosis induced by radiotherapy in combination with α-bisabolol (**A**) Apoptotic rate of RL95-2. The RL95-2 was treated with α-bisabolol (4 μmol/l), radiotherapy (4 Gy) or the combination of α-bisabolol and radiotherapy, respectively, and then was analyzed by Hoechst 33258 staining. The apoptotic cells were marked with white arrows. Scale bar = 50 μm. (**B**) Western blot for crucial proteins in XIAP/Caspase-3 pathway. GAPDH was used as the loading control. Three experiments were performed independently, and ±STDEV was shown with each value, *P<0.05 and **P<0.01.

To investigate its molecular mechanism, we detected caspase-3 and its inhibitor, XIAP. The results indicated that caspase-3 was markedly increased as the decrease in XIAP (Figure 4B), which suggested the increase in apoptosis was mediated by by XIAP/caspase-3 pathway. To confirm this hypothesis, we detected downstream proteins (PARP, cleaved PARP and COX-2) of caspase-3. As our expected, the COX-2 and cleaved PARP were significantly reduced and increased, respectively. However, the expression of PARP showed no change in our study (Figure 4B).

## Discussion

EC is a major threat to women’s health and gets wide attention [2,4]. Although the survival rate of patients is relatively high if EC is diagnosed in early stages, it can be very lethal and recur frequently after surgery when it develops into advanced stages. For the preoperative evaluation or clinical management of EC, the magnetic resonance imaging (MRI) and hysteroscopic excisional biopsy (HEB) were employed usually, and combining MRI and HEB could elevate the accuracy in identifying low-risk patients [39]. Besides, the laparoscopy might also become a useful method to manage early stage EC, in which it exhibited advantageous in operative morbidity and hospital stay over laparotomy [40].

Radiotherapy is an efficient mothed employed widely to inhibit EC cells and reduce this risk after surgery, while the radioresistance of EC limits its effect. Therefore, to improve the efficacy of radiotherapy on EC, many drugs are identified with synergistic effect and can be used as adjuvant treatments. α-bisabolol is well-known for its anti-inflammatory and anti-carcinoma functions in various cancers [27,28]. However, its effect on EC and the potential as an adjuvant drug in radiotherapy is still unknown.

In the present study, we found significant anti-cancer effect of α-bisabolol on EC cells. It is demonstrated by our results that EC cells are more sensitive to the killing effect of α-bisabolol than normal endometrial cells in the concentration ranging from 4 to 16 μmol/l. With the appropriate concentration (4 μmol/l), the ability of EC cells for migration and invasion were also markedly reduced by α-bisabolol. Thus, it is concluded from these inhibitory effects of α-bisabolol on the proliferation, migration and invasion of EC cells that α-bisabolol may be a promising anti-carcinoma drug for EC.

Inspired by its anti-cancer effect, we next investigated its effect in radiotherapy. Clonogenic assays revealed that, by using α-bisabolol, the formation of EC colonies were significantly suppressed though the inhibitory effect of α-bisabolol is weaker than that of irradiation. It was also shown the viability rate, EC_50_ and LC_50_ of EC cells were reduced when α-bisabolol was used, suggesting the increased effect of radiotherapy may be because α-bisabolol sensitizes EC cells. This conclusion was further demonstrated by the decrease in MMP-9 and cyclin E. MMP-9 and cyclin E both are famous biomarkers of cancers, which perform a lot of biological functions related to tumorigenesis. Their expressions are positively related to histologic grade, invasion and resistance of tumors. The stable expression of cyclin E when only using α-bisabolol or radiotherapy may be due to the compensation effect of other molecular pathway [41–43] or the low dose we used, while it was significantly reduced when using α-bisabolol and radiotherapy together. Thus, the decrease we detected indicated that EC cells were suppressed, and the progression of EC was slowed by the combination of α-bisabolol and radiotherapy.

Cell apoptosis may play a key role in many diseases, such as endometriosis. Its inhibition in endometriotic cells, in which the expression of anti-apoptotic gene B-cell lymphoma 2 (Bcl-2) may get activated [44], and activation in peritoneal fluid mononuclear cells may create a permissive microenvironment for the progression of endometriosis [45]. According to our results, EC has strong resistance to the apoptosis induced by α-bisabolol or radiotherapy. However, by using radiotherapy in combination with α-bisabolol, the apoptotic rate of EC cells was nearly doubled. Our detection of apoptosis-related proteins exhibited the significant decrease in XIAP, one type of the inhibitor of apoptosis proteins, and the activation of caspase-3 pathway, which respond to the apoptotic execution. It was further demonstrated by detecting the expression of downstream effectors of caspase-3. COX-2 was reduced, and Cleaved-PARP was markedly increased, which indicated the activation of apoptotic pathway mediated by caspase-3. Interestingly, the protein level of PARP was not down-regulated, although PARP was cleaved by caspase-3. This result may suggest that the Cleaved-PARP can be a more reliable biomarker for apoptosis than PARP itself.

Altogether, in our study, α-bisabolol exhibited the strong inhibitory activity on EC cells and enhanced the radiosensitivity of EC cells during radiotherapy. Although more clinical experiments are needed, it offered a new alternative for overcoming the radioresistance of EC. It was also demonstrated in our research that α-bisabolol could increase apoptosis via XIAP/caspase-3 pathway in radiotherapy. For further understanding how α-bisabolol regulates apoptosis in EC cells, its further molecular pathways that regulate XIAP/caspase-3 pathway are needed to be explored in the future.

## Abbreviations

DMEM: Dulbecco’s modified Eagle’s medium
EC: endometrial cancer
EC_50_: half-maximal effective concentration
HEB: hysteroscopic excisional biopsy
LC_50_: half-maximal lethal concentration
MMP-9: matrix metalloproteinase-9
MRI: magnetic resonance imaging
TBST: TBS with 0.05% Tween 20
XIAP: X-linked inhibitor of apoptosis protein
